# Elevated intracranial dopamine impairs the glutamate-nitric oxide-cyclic guanosine monophosphate pathway in cortical astrocytes in rats with minimal hepatic encephalopathy

**DOI:** 10.3892/mmr.2014.2386

**Published:** 2014-07-16

**Authors:** SAIDAN DING, WEILONG HUANG, YIRU YE, JIANJING YANG, JIANGNAN HU, XIAOBIN WANG, LEPING LIU, QIN LU, YUANSHAO LIN

**Affiliations:** 1 Zhejiang Provincial Key Laboratory of Aging and Neurological Disease Research, Department of Surgery Laboratory, The First Affiliated Hospital of Wenzhou Medical University, Wenzhou, Zhejiang 325000, P.R. China; 2 Neurosurgery Department, The First Affiliated Hospital of Wenzhou Medical University, Wenzhou, Zhejiang 325000, P.R. China; 3 Department of Computer, Wenzhou Medical University, Wenzhou, Zhejiang 325000, P.R. China; 4 First Department of Neurology, The First Affiliated Hospital of Wenzhou Medical University, Wenzhou, Zhejiang 325000, P.R. China

**Keywords:** dopamine, primary cortical astrocytes, glutamate-nitric oxide-cyclic guanosine monophosphate, minimal hepatic encephalopathy

## Abstract

In a previous study by our group memory impairment in rats with minimal hepatic encephalopathy (MHE) was associated with the inhibition of the glutamate-nitric oxide-cyclic guanosine monophosphate (Glu-NO-cGMP) pathway due to elevated dopamine (DA). However, the effects of DA on the Glu-NO-cGMP pathway localized in primary cortical astrocytes (PCAs) had not been elucidated in rats with MHE. In the present study, it was identified that when the levels of DA in the cerebral cortex of rats with MHE and high-dose DA (3 mg/kg)-treated rats were increased, the co-localization of *N*-methyl-d-aspartate receptors subunit 1 (NMDAR1), calmodulin (CaM), nitric oxide synthase (nNOS), soluble guanylyl cyclase (sGC) and cyclic guanine monophosphate (cGMP) with the glial fibrillary acidic protein (GFAP), a marker protein of astrocytes, all significantly decreased, in both the MHE and high-dose DA-treated rats (P<0.01). Furthermore, NMDA-induced augmentation of the expression of NMDAR1, CaM, nNOS, sGC and cGMP localized in PCAs was decreased in MHE and DA-treated rats, as compared with the controls. Chronic exposure of cultured cerebral cortex PCAs to DA treatment induced a dose-dependent decrease in the concentration of intracellular calcium, nitrites and nitrates, the formation of cGMP and the expression of NMDAR1, CaM, nNOS and sGC/cGMP. High doses of DA (50 μM) significantly reduced NMDA-induced augmentation of the formation of cGMP and the contents of NMDAR1, CaM, nNOS, sGC and cGMP (P<0.01). These results suggest that the suppression of DA on the Glu-NO-cGMP pathway localized in PCAs contributes to memory impairment in rats with MHE.

## Introduction

Minimal hepatic encephalopathy (MHE) refers to the subtle changes in cognitive function, electrophysiological parameters, cerebral neurochemical/neurotransmitter homeostasis, cerebral blood flow, metabolism and fluid homeostasis that are observed in patients with cirrhosis, who have no clinical evidence of hepatic encephalopathy (1). The glutamate-nitric oxide-cyclic guanine monophosphate (Glu-NO-cGMP) pathway is involved in certain types of learning and memory (2,3). Activation of *N*-methyl-d-aspartate receptors subunit 1 (NMDAR1) by glutamate increases calcium in postsynaptic neurons. Calcium binds to calmodulin (CaM) and activates neuronal nitric oxide synthase (nNOS), increasing NO, which activates soluble guanylyl cyclase (sGC), increasing cyclic guanine monophosphate (cGMP), part of which is released to the extracellular space and is functionally important in learning and memory (2). A previous study by our group (4) identified that a catechol-O-methyltransferase (COMT) inhibitor, a protein involved in the accumulation of dopamine (DA), was upregulated in cirrhotic livers in rats with MHE by 2-dimensional gel electrophoresis/mass spectrometry (2-DE/MS). Furthermore, the levels of DA in cirrhotic livers, serums and the hippocampi in the MHE group were notably increased, and the Glu-NO-cGMP memory pathway in hippocampal neurons was inhibited by the elevation of DA *in vivo* and *in vitro*. Therefore, it was hypothesized that the pathogenesis of MHE may be associated with the elevation in DA characteristic of cirrhotic livers. Furthermore, the study demonstrated that the DA levels were increased in cirrhotic livers and that it crossed the blood-brain barrier, migrated into the brains of rats with MHE and inhibited their learning and memory ability by blocking the Glu-NO-cGMP pathway in neurons (4). However, whether astrocytes were involved in the pathogenesis of MHE remained elusive.

One type of astrocyte, expressing glutamate receptors, responds to the synaptic release of glutamate via channel-mediated currents and is involved in the function of the Glu-NO-cGMP pathway. Activation of mGluR3 receptors in striatal neurons (5), hippocampal neurons (6), cerebellar granule cell neurons (7) and rat cerebellar astrocytes (8) is accompanied by a reduction in the levels of cyclic adenosine monophosphate (cAMP). In the majority of tissues, NO acts as an intracellular signaling molecule and is formed in all brain cells, including astrocytes, by NOS from l-arginine (9). The major physiological receptor for NO is sGC, an αβ heterodimer that catalyses the conversion of guanosine triphosphate (GTP) to cGMP and which acts as a secondary messenger, modulating the activity of cGMP-dependent protein kinases, cyclic nucleotide phosphodiesterases and cyclic nucleotide-gated channels (10). Several studies have suggested that astrocytes integrate learning and memory in the cerebral cortex by having a direct role in the modulation of synaptic plasticity and long-term potentiation (11).

The present study delineated the role of the Glu-NO-cGMP pathway localized in astrocytes in MHE-associated memory loss, particularly focusing on the effect of elevated DA from cirrhotic liver in the brains of an MHE *in vivo* model.

## Materials and methods

### MHE models and treatments

A total of 50 Sprague-Dawley rats (Experimental Animal Center of The Chinese Academy of Sciences in Shanghai, Shanghai, China) weighing 220–250 g were used. The present study was approved by the ethics committee of the First Affiliated Hospital of Wenzhou Medical University (Wenzhou, China) regarding the care and use of animals for experimental procedures. Rats were housed under controlled conditions of temperature (24±1°C) and light (12 h light starting at 07:00 am). Prior to the experimental stage, all animals were subject to a series of behavioral tests including Y-maze (YM), open-field (OF), elevated-plus maze (EPM) and water-finding task (WFT) tests. There was a 15 min interval between each behavioral test for each rat. The normalized values of these behavioral tests were obtained. Rats were then randomly divided into two groups; the control group (n=20) and the thioacetamide (TAA) group (n=30). MHE was induced by intraperitoneal injection (i.p.) of TAA (200 mg/kg in normal saline; Sigma-Aldrich, St. Louis, MO, USA) twice a week for a period of eight weeks. Then, the rats were subjected to the same behavioral tests again. Rats included in the MHE group were required to meet the following criteria: i) The values of one of the behavioral tests in the MHE group being significantly different from those of the control group and ii) the EEG revealing no typical slow wave of hepatic encephalopathy (12). At 24 h following MHE induction, NMDA (0.3 mM) was also administered to the rats for 30 min by intraperitoneal injection. Liver, serum and cerebral cortex were collected for fluorescent staining, immunoblotting and determination of DA.

### DA-injected rat models and treatments

Rats were administered DA hydrochloride (0.3 and 3 mg/kg; Sigma-Aldrich) by i.p. injection twice per week for four weeks. All of the rats were subjected to the OF, YM, EPM and WFT tests. Following the final injection, NMDA (0.3 mM; Sigma-Aldrich) was also administered to the rats for 30 min by intraperitoneal injection. Liver, serum and cerebral cortex specimens were collected for fluorescent staining, immunoblotting and determination of DA.

### Behavioral tests

The OF test was performed as previously described (13). Briefly, rats were individually placed at the center of a 10×10 cm gray plastic field (with 20 cm interval black grids) surrounded by a 20-cm wall and allowed to move freely for 3 min. Ambulation was measured and defined as the total number of grid line crossings (13).

The apparatus for the YM test was composed of gray plastic, with each arm being 40 cm long, 12 cm high, 3 cm wide at the base and 10 cm wide at the top. The three arms were connected at an angle of 120°. Rats were individually placed at the end of one arm and allowed to explore the maze freely for 8 min. Total arm entries and spontaneous alternation percentage (SA%) were measured. SA% was defined as the ratio of the arm choices that differed from the previous two choices (‘successful choices’) to the total choices during the run (‘total entry minus two’ because the first two entries were not evaluated). For example, if a mouse made 10 entries, such as 1-2-3-2-3-1-2-3-2-1, there were 5 successful choices in 8 total choices (10 entries minus 2; 13,14).

The EPM test apparatus was composed of four crossed arms. Two arms were open (50×10 cm grey plastic floor plate without walls), whereas the other two were closed (same floor plates with 20 cm-high transparent acrylic wall). The maze was set at a height of 100 cm above the floor. Rats were allowed to explore the maze freely for 90 sec. The parameters that were examined were as follows: (i) The transfer latency (the time elapsed until the first entry to a closed arm); (ii) the duration of the first stay in a closed arm (the time from the first entry to a closed arm to the first escape from the arm) and (iii) the cumulative time spent in the open/closed arms (13,15).

The WFT test was performed to analyze latent learning or retention of spatial attention ability in the rats. The testing apparatus consisted of a grey plastic rectangular open field (50×30 cm, with a black 10 cm^2^ grid) with a 15 cm high wall and a cubic alcove (10×10×10 cm), which was attached to the center of one longer wall. A drinking tube was inserted through a hole at the center of the alcove ceiling, with the tip of the tube placed at 5 cm for training or at 7 cm for the trial from the floor. A mouse was first placed at the near-right corner of the apparatus and allowed to explore freely for 3 min. Rats were excluded from the analysis when they were not able to locate the tube within the 3 min exploration. Following completion of the training, the rats were deprived of water for 24 h. In the trial session, rats were again individually placed at the same corner of the apparatus and allowed to locate and drink the water in the alcove. The elapsed time until the first entry into the alcove (entry latency, EL), until the first touching, sniffing or licking of the water tube (contacting latency, CL) and until the initiation of drinking from the water tube (drinking latency, DL) were measured (13,16,17).

### Histopathology

Liver tissues were ﬁxed in 10% formalin for 24 h and then parafﬁn-embedded in an automated tissue processor; 5 μm sections were stained with hematoxylin and eosin (H&E) or Sirius red and subjected to histopathological examination.

### Determination of DA levels

A total of 300–800 μl of 0.4 M HClO_4_ solution containing 0.1% (w/v) Na_2_S_2_O_5_ was added to the liver, serum or cerebral cortex samples, and the mixture was homogenized by sonication (Labsonic U; B. Braun Biotech International Gmbh, Melsungen, Germany). The homogenates were centrifuged for 15 min at 20,000 × g at 4°C and aliquots of the supernatants were obtained for analysis of DA using a high performance liquid chromatography (HPLC) technique (E2695; Waters, Inc., Milford, MA, USA) (18).

### Double-labeled fluorescent staining of cerebral cortex sections

Four-micron frozen cerebral cortex sections fixed in acetone or 4% formaldehyde were blocked for endogenous peroxidase activity with 0.03% H_2_O_2_ if appropriate. Blocking was achieved with phosphate-buffered saline (PBS) containing 5% normal goat serum (Wuhan Boster Biological Technology, Ltd., Wuhan, China) for 1 h at room temperature. Sections were then incubated overnight at 4°C with the following primary antibodies; NMDAR1 (1:100; mouse monoclonal; Abcam, Cambridge, MA, USA), CaM (1:100; mouse monoclonal; Abcam), nNOS (1:50; Rabbit monoclonal; Abcam), sGC (1:50; rabbit polyclonal; Abcam), cGMP (1:50; mouse monoclonal; Santa Cruz Biotechnology, Inc., Santa Cruz, CA, USA) and GFAP (1:50; rabbit polyclonal/mouse monoclonal; Abcam). Binding of primary antibodies was detected by incubating the sections for 30 min with fluorescein isothiocyanate (FITC) (green)/Alexa Fluor 594 (red) conjugated secondary antibody. Imaging was performed with a Leica TCS SP2 confocal laser scanning microscope (Leica Microsystems, Wetzlar, Germany). The image data were analyzed and quantified using ImagePro Plus software 6.0 (Media Cybernetics, Inc., Rockville, MD, USA).

### Isolation of astrocytes

Primary cortical astrocytes (PCAs) were prepared from one-day-old Sprague-Dawley rat pups (19). Tissues of cerebral cortex were dissociated into a cell suspension using mechanical digestion. Cells were plated in 75 cm^2^ tissue culture flasks at a concentration of 15×10^6^ cells in 11 ml medium and incubated for 72 h. The medium was changed at this time-point and every 72 h. Following incubation of the primary cultures for seven days, the medium was changed completely (11 ml) and the caps were tightened. Flasks were wrapped in plastic, placed on a shaker platform in a horizontal position with the medium covering the cells and centrifuged at 200 × g for 18 h at 37°C to separate the oligodendrocytes from the astrocytes. The contents were then poured into a new 75 cm^2^ flask and incubated for seven days. Following this, the cells were plated in poly-l-lysine-precoated six-well plates, incubated with DA (final concentrations of 5 or 50 μM) in 1% serum-containing DMEM/F12 medium for 24 h. Then, 0.3 mmol/l NMDA was added and the incubation continued for another 5 min.

### Changes in intracellular Ca^2+^ in PCAs

The changes in intracellular Ca^2+^ were monitored in single PCAs by confocal microscopy using Fluo-3/AM as previously described (20).

### Determination of nitrites and nitrates

The levels of nitrites and nitrates were measured in PCAs utilizing the Griess method with nitrate reductase (21). A total of 100 μl of the culture supernatant was mixed with equal volumes of Griess reagent. Following 10 min at 20–25°C absorbance was measured at 540 nm.

### Determination of cGMP levels

The ELISA assay for the quantitative determination of cGMP in PCAs was then performed using cGMP fluorescent assay kits (Molecular Devices Co., Inc., Sunnyvale, CA, USA).

### Fluorescent staining of PCAs

PCAs were seeded and cultured on glass coverslips precoated with 0.01% poly-l-lysine (Sigma-Aldrich) for 1 h. Following treatment of the cells with DA (final concentration of 5 or 50 μM) for 24 h, they were fixed with 4% paraformaldehyde for 30 min and then treated with 0.1% Triton X-100 for 10 min at room temperature.

Blocking was achieved with PBS containing 5% normal goat serum for 1 h at room temperature. Sections were then incubated overnight at 4°C with the following primary antibodies: NMDAR1 (1:100; Abcam), CaM (1:100; Abcam), nNOS (1:50; Abcam), sGC (1:50; Abcam) and cGMP (1:50; Santa Cruz Biotechnology, Inc.). Binding of primary antibodies was detected by incubating the sections for 30 min with Alexa Fluor 594 (red) conjugated secondary antibody. Imaging was performed with a Leica TCS SP2 confocal laser scanning microscope (Leica Microsystems). The image data were analyzed and quantified using ImagePro Plus software (Media Cybernetics, Inc.) (22).

### Immunoblotting of PCAs

PCAs were harvested in a lysis buffer [50 mM Tris HCl (pH 7.4), 150 mM NaCl, 1% Triton X-100 and protease inhibitors (Sigma-Aldrich)]. The total amount of protein was determined by the bicinchoninic acid protein assay (Amresco, Solon, OH, USA). Samples (50 μg protein) were separated by 10% SDS-PAGE and electroblotted to polyvinylidene fluoride membranes, which were blocked by incubation in 5% non-fat milk powder dissolved in TBS-T (150 mM NaCl, 50 mM Tris and 0.05% Tween-20). Following transfer, proteins were probed using a primary antibody; NMDAR1 (1:1000; Cell Signaling Technology, Inc.), CaM (1:1000; Abcam), nNOS (1:1500; Abcam), sGC (1:1000; Abcam) and cGMP (1:200, Santa Cruz Biotechnology). Then, horseradish peroxidase-conjugated secondary antibody was used. Following extensive washing, protein bands detected by antibodies were visualized by enhanced chemiluminescence reagent (Pierce Biotechnology, Inc., Rockford, IL, USA) following exposure on Kodak BioMax film (Kodak, Rochester, NY, USA). The films were subsequently scanned and the band intensities were quantified using Quantity One software (Bio-Rad Laboratories, Inc., Hercules, CA, USA).

### Statistical analysis

A two-tailed Student’s t-test was used to determine the statistical significance of difference in values between the control and experimental preparations. All data are presented as the mean ± standard deviation. P<0.05 or P<0.01 were considered to indicate a statistically significant difference between values.

## Results

### Memory impairment and elevation of intracranial DA levels in MHE models

H&E and Sirius red staining in the livers of TAA-treated rats revealed inflammatory cell infiltration around the portal area, with collagen deposition or fibrous septa formation (Fig. 1A and B), suggesting that the liver ﬁbrosis model was successfully established.

Rats were then subjected to a series of behavioral tests, including OF, YM, EPM and WFT tests. There were significant differences in the voluntary activities in the OF test between the MHE and control groups following treatment (Fig. 1C). The SA% in the YM of the TAA-treated rats was significantly decreased (P<0.01), compared with that of the control rats (Fig. 1D). In the EPM test, TAA-treated rats remained in the open arms for significantly longer than in the closed arms, as compared with the controls (Fig. 1E). In the WFT test, significant delays in EL, CL and DL were detected in the TAA-treated rats as compared with the controls (Fig. 1F). In the EEG tests, 6/25 TAA-treated rats exhibited slow wave (Theta =4–7 Hz or Delta <4 Hz wave; Fig. 1G). Therefore, the incidence of MHE in the TAA group was 76.0% (19/25).

Considering that the increased levels of DA in the liver (Fig. 1H), serum (Fig. 1I) and cerebral cortex (Fig. 1J) of MHE rats were observed in a previous study by our group (4), the present study examined whether the concentration of DA in the liver, serum and cerebral cortex of rats with MHE would exhibit similar trends. The data were consistent with those of the previous study, confirming the earlier results (Fig. 1H). The results confirmed that DA, when elevated in the liver, crossed the blood-brain barrier and permeated into the brains of rats with MHE, as previously observed.

### Confirmation of memory impairment caused by elevation of intracranial DA

To confirm whether memory impairment in rats with MHE was associated with DA transported into the brain, normal rats were subjected to an i.p. injection of DA (low dose, 0.3 mg/kg and high dose, 3 mg/kg). At a week following the injection, all rats were again subjected to behavioral tests, including OF, YM, EPM and WFT tests. The mean voluntary activities in the OF test were significantly increased following high-dose DA treatment (Fig. 2A). The SA% (P<0.01) in the YM test was significantly decreased in high-dose DA-treated rats (Fig. 2B). In the EPM test, the high-dose DA-treated rats remained in the open arms for significantly longer and spent a shorter time in the closed arms as compared with the controls (Fig. 2C). In the WFT, EL, CL and DL tests, the responses were significantly delayed in the high-dose DA-treated rats as compared with the controls (Fig. 2C). The control and DA-treated rats demonstrated an Alpha (8–13 Hz) band in the EEG tests (Fig. 2E).

It was also observed that the levels of DA in the serum (Fig. 2F) and cerebral cortex (Fig. 2G) were significantly elevated following treatment with a high dose of DA (P<0.01), confirming that when blood levels were high, DA crossed the blood-brain barrier, permeated the brains and subsequently attenuated cognitive function in rats.

### Inactivation of Glu-NO-cGMP pathway in astrocytes of the cerebral cortex by DA in vivo

A previous study by our group identified that memory impairment in rats with MHE was associated with the inactivation of the Glu-NO-cGMP pathway in neurons by high doses of DA in the brain (4). Therefore, the present study examined whether the inactivation of the Glu-NO-cGMP pathway in astrocytes contributed to memory impairment in rats with MHE. The proteins of the Glu-NO-cGMP pathway (NMDAR1, CaM, nNOS, sGC and cGMP) were co-localized with GFAP in the cerebral cortex. The co-localization indicated that the four proteins were significantly decreased in the rats with MHE, as compared with the normal rats (Fig. 3A–E), indicating that the inhibition of the Glu-NO-cGMP pathway in astrocytes of rats with MHE was associated with memory impairment. As expected, the NMDAR1, CaM, nNOS, sGC and cGMP levels were substantially increased following i.p. injection of NMDA (Fig. 3E). The augmentation of NMDAR1, CaM, nNOS, sGC and cGMP levels induced by NMDA was inhibited in rats with MHE (Fig. 3A–E).

Following this, it was determined whether DA was involved in the inhibition of the Glu-NO-cGMP pathway in astrocytes in the DA (0.3 and 3 mg/kg)-treated rats. DA treatment also induced a dose-dependent decrease in the expression of the four proteins localized in the astrocytes of the cerebral cortex of rats. The co-localization demonstrated that the four proteins were highly expressed in the astrocytes of normal and low-dose DA-treated rats and weakly expressed in the astrocytes of high-dose DA-treated rats (Fig. 4A–E), indicating high-dose DA-induced inhibition of the Glu-NO-cGMP pathway in the astrocytes of the cerebral cortex of rats. Furthermore, it was identified that high-dose DA (3 mg/kg) decreased NMDA-mediated augmentation of NMDAR1, CaM, nNOS, sGC and cGMP expression levels in astrocytes (Fig. 4A–E).

### Inactivation of the Glu-NO-cGMP pathway in PCAs by DA

To confirm the inhibition of the activation of the Glu-NO-cGMP pathway by DA in PCAs, the levels of intracellular Ca^2+^, nitrites and nitrates and cGMP in DA-treated PCAs were assessed. NMDA (0.3 mmol/l) was added to the normal and DA-treated PCAs. As revealed in Fig. 5Aa, NMDA induced increases in calcium levels in normal PCAs. Chronic exposure to high-dose DA significantly decreased NMDA-induced increases in calcium (Fig. 5Ad). Basal concentrations of nitrites and nitrates were lower in high-dose DA-treated PCAs (1.15±0.89 mol/l) than in the controls (2.51±0.56 mol/l) (Fig. 5B). NMDA increased the levels of nitrites and nitrates in the control PCAs. NMDA-induced elevation of NO was also impaired in DA-treated PCAs (Fig. 5B).

DA treatment induced a dose-dependent decrease in the formation of cGMP in PCAs. As shown in Fig. 5C, the content of basal cGMP in PCAs following low-dose DA treatment (5 μM) revealed no difference compared with those of the controls. Chronic exposure to high levels of DA significantly decreased the basal cGMP concentration. The addition of NMDA increased cGMP levels in the control PCAs, 5 and 50 μM DA-treated PCAs to 12.31±2.02, 11.79±1.84 and 6.53±1.12 pmol/mg protein, respectively (Fig. 5C), indicating a significant reduction of 38% for 50 μM DA treatment in the function of the Glu-NO-cGMP pathway.

Following this, the effect of DA on the expression of proteins of the Glu-NO-cGMP pathway was confirmed by immunostaining and immunoblot analysis of NMDAR1, CaM, nNOS, sGC and cGMP in PCAs. DA treatment induced a dose-dependent decrease in the expression of the four proteins in PCAs. The results of the immunoblotting analyses revealed that the expression of the four proteins was downregulated in PCAs exposed to high-dose DA (50 μM) as compared with the control group (Fig. 6A). As demonstrated in Fig. 6B, immunofluorescent assessment revealed that low-dose DA treatment (5 μM) failed to attenuate the number of NMDAR1, CaM, nNOS or sGC immunoreactive PCAs. By contrast, the high-dose DA treatment (50 μM) successfully decreased the expression of the four proteins. The addition of NMDA upregulated the expression of the four proteins in PCAs, which was an effect that was inhibited by high-dose DA (Fig. 6A and B). These results suggested that DA inhibits the function of the whole Glu-NO-cGMP pathway.

## Discussion

In the present study, it was demonstrated that chronic stimulation of astrocytes in the cerebral cortex by toxic DA significantly deteriorated the expression of proteins involved in the Glu-NO-cGMP pathway. The results revealed that chronic exposure to DA affected the Glu-NO-cGMP pathway in astrocytes of the rat cerebral cortex *in vivo* at different stages. Exposure to DA significantly reduced the levels of NMDAR1, CaM, nNOS, sGC and cGMP (Fig. 3) and the activation of NMDAR1, CaM, nNOS, sGC and cGMP by NMDA (Fig. 1). This effect may subsequently contribute to the reduced formation of cGMP. Therefore, the present study provided the first evidence, to the best of our knowledge, suggesting that the Glu-NO-cGMP pathway localized in astrocytes may be important in the pathogenesis of DA-associated memory impairment in rats with MHE.

Chronic exposure of rats to DA appeared to affect the Glu-NO-cGMP pathway at different stages. A number of studies have suggested that high concentrations of DA reduce NMDAR1-mediated currents and postsynaptic potentials in pyramidal neurons (23–25). Another recent study reported that the direct inhibition of NMDAR1 by D1 ligands (DA) is due to the blockade of the channel pore (26). Several previous studies have demonstrated that DA inhibits NMDA receptor-mediated nNOS stimulation, and thus has a role in nNOS-NO signaling in the generation of striatal cGMP (27–33). NO is partially controlled by nigrostriatal DA input and affects striatal functions (34–37). One study suggested that the parkinsonian state is associated with an abnormal NO/sGC cascade. The DA-deprived striatum revealed a reduction in the standard NO-mediated inhibition (38). The present study demonstrated that the decreased content of NMDAR1, CaM, nNOS, sGC and cGMP, and the impairment of NMDA-induced activation of NMDAR1, CaM, nNOS, sGC and cGMP occurred in astrocytes treated with high concentrations of DA, suggesting that DA was responsible for impaired activation of any of the proteins of the Glu-NO-cGMP pathway and was involved in the impairment of cognitive ability.

In conclusion, the present study provided evidence for a novel theory accounting for memory dysfunction in MHE. The results demonstrated that high DA levels in cirrhotic livers led to elevated DA levels in the brains of MHE models, and that the subsequent DA-dependent inactivation of the Glu-NO-cGMP pathway in astrocytes triggered memory impairment in the rats with MHE. The effect of DA on the impairment of the Glu-NO-cGMP pathway in astrocytes provided new insights that facilitate the understanding of the function of astrocytes. These results provided evidence of not only a novel pathological hallmark of MHE but also a candidate target for MHE therapy. Further investigations should focus on the downstream cascades of the Glu-NO-cGMP pathway that may also be involved in DA-induced memory impairment in MHE.

## Figures and Tables

**Figure 1:** Memory impairment and elevated DA in MHE models. (A) Hematoxylin and eosin (scale bar, 50 μm) and (B) Sirius red staining (scale bar, 100 μm) of liver sections from the control and TAA-treated rats. (C) Ambulation in open-field test of the control and TAA-treated rats (left, pretreatment; right, eight-week treatment). (D) SA% in YM of the control and TAA-treated rats (left, pretreatment; right, 8-week treatment). (E) Results of EPM (TL, transfer latency; first stay, duration of the first stay; open, time spent in the open arms; closed, time spent in the closed arms). (F) Results of the WFT test (EL, entry latency; CL, contacting latency; DL, drinking latency). (G) The cerebral signal of rats observed in the scalp EEG falls in the Alpha (8–13 Hz) range in the control and MHE rats. Levels of DA in (H) the liver, (I) serum and (J) cerebral cortex analyzed in the control and MHE groups. Data are presented as the mean ± standard deviation. ^*^P<0.05, ^**^P<0.01 vs. control treatment by Dunnett’s post-hoc test. DA, dopamine; MHE, minimal hepatic encephalopathy; YM, Y-maze; SA%, spontaneous alternation percentage; EPM, elevated-plus maze; WFT, water-finding task; TAA, thioacetamide.

**Figure 2:** Effect of intracranial elevated DA on memory impairment. (A) Ambulation in OF of control and DA (0.3 and 3 mg/kg)-treated rats (left, pretreatment; right, eight-week treatment). (B) SA% in YM of control and DA (0.3 and 3 mg/kg) -treated rats (left, pretreatment; right, eight-week treatment). (C) Results of EPM (TL, transfer latency; first stay, duration of the first stay; open, time spent in the open arms; closed, time spent in the closed arms). (D) Results of WFT (EL, entry latency; CL, contacting latency; DL, drinking latency). (E) No Theta (4–7 Hz) or Delta (<4 Hz) bands (slow wave) were observed in EEG of DA-treated rats. Levels of DA in the (F) serum and (G) cerebral cortex analyzed in the control and DA-treated groups. Data are presented as the mean ± standard deviation. ^*^P<0.05, ^**^P<0.01 vs. control treatment by Dunnett’s post-hoc test. DA, dopamine; MHE, minimal hepatic encephalopathy; OF, open-field; YM, Y-maze; SA%, spontaneous alternation percentage; EPM, elevated-plus maze; WFT, water-finding task; EEG, electroencephalogram.

**Figure 3:** The Glu-NO-cGMP pathway was inactivated in astrocytes of cerebral cortex in MHE models. (A) Co-localization of NMDAR1, (B) CaM, (C) nNOS, (D) sGC, (E) cGMP (green) with GFAP (an astrocytic marker, red) is indicated by the overlap of signals resulting in yellow staining in the cerebral cortex of the control and MHE rats with the absence or the presence of NMDA (0.3 mM) (scale bar, 25 μm). Glu-NO-cGMP, glutamate-nitric oxide-cyclic guanosine monophosphate; MHE, minimal hepatic encephalopathy; NMDAR1, *N*-methyl-d-aspartate receptors subunit 1; CaM, calmodulin; nNOS, nitric oxide synthase; sGC, soluble guanylyl cyclase; cGMP, cyclic guanine monophosphate; GFAP, glial fibrillary acidic protein.

**Figure 4:** The Glu-NO-cGMP pathway was inhibited by DA (0.3 and 3 mg/kg) in astrocytes of the cerebral cortex *in vivo*. Double immunofluorescent staining of cerebral cortex of control and DA (0.3 and 3 mg/kg) -treated rats with the absence or the presence of NMDA using antibodies against GFAP (red) and (A) NMDAR1, (B) CaM, (C) nNOS, (D) sGC and (E) cGMP (green) (scale bar, 25 μm). Glu-NO-cGMP, glutamate-nitric oxide-cyclic guanosine monophosphate; NMDAR1, *N*-methyl-d-aspartate receptors subunit 1; DA, dopamine; CaM, calmodulin; nNOS, nitric oxide synthase; sGC, soluble guanylyl cyclase; cGMP, cyclic guanine monophosphate; GFAP, glial fibrillary acidic protein.

**Figure 5:** The function of the Glu-NO-cGMP pathway is impaired in PCAs chronically exposed to DA. (A) Free intracellular Ca^2+^ content was followed with fluo-3/AM using confocal microscopy. The basal Ca^2+^ levels were recorded for 200 sec, then 0.3 mM NMDA was added and the fluorescence was recorded for 1,600 sec. Typical traces are demonstrated in (Aa), (Ab) and (Ac). The increase in calcium at 1,600 sec compared with 200 sec was similar in (Aa) the control astrocytes or (Ab) DA-treated astrocytes. The values (mean ± SD) of quadruplicate samples from six different cultures are illustrated in (Ad), ^**^P<0.01 vs. controls. (B) The levels of nitrites under basal conditions, 5 min following the addition of 0.3 mM NMDA. The values were significantly different (P<0.05) from basal nitrites prior to the addition of NMDA, and are indicated by (i) for control astrocytes and by (ii) and (iii) for 5 μM and 50 μM DA-treated astrocytes, respectively. Values that are signiﬁcantly different in astrocytes exposed to ammonia from the control astrocytes are indicated by asterisks, ^**^P<0.01 vs. controls. (C) The content of cGMP in astrocytes treated or not (basal) with NMDA (0.3 mM) was measured. Values are the presented as the mean ± SD of triplicate samples from seven different cultures. Values that were signiﬁcantly different (P<0.05) from basal cGMP prior to the addition of NMDA are indicated by (i) for the control astrocytes and by (ii) and (iii) for the astrocytes exposed to 5 μM DA and 50 μM DA, respectively. Values that are signiﬁcantly different in astrocytes exposed to DA from control astrocytes are indicated by asterisks, ^**^P<0.01 vs. controls. PCAs, primary cortical astrocytes; DA, dopamine; Glu-NO-cGMP, glutamate-nitric oxide-cyclic guanosine monophosphate; NMDA, *N*-methyl-d-aspartate; cGMP, cyclic guanine monophosphate; SD, standard deviation.

**Figure 6:** The effect of DA (5 and 50 μM) on the Glu-NO-cGMP pathway in PCAs. (A) Immunoblot analysis of PCAs treated with DA (5 and 50 μM). Expression of NMDAR1, CaM, nNOS, sGC and cGMP was normalized to the corresponding GAPDH protein. Data are presented as the mean ± standard deviation. The values were signifcantly different (P<0.05) from basal nitrites prior to the addition of NMDA and are indicated by (i) for control astrocytes and by (ii) and (iii) for 5 μM and 50 μM DA-treated astrocytes, respectively. ^*^P<0.05, ^**^P<0.01 vs. the control group. (B) Immunofluorescence staining of DA (5 and 50 μM)-treated PCAs in the absence or the presence of NMDA (0.3 mM) using the anti-NMDAR1, CaM, nNOS, sGC and cGMP antibodies (scale bar, 50 μm). PCAs, primary cortical astrocytes; DA, dopamine; NMDAR1, *N*-methyl-d-aspartate receptors subunit 1; Glu-NO-cGMP, glutamate-nitric oxide-cyclic guanosine monophosphate; CaM, calmodulin; nNOS, nitric oxide synthase; sGC, soluble guanylyl cyclase; cGMP, cyclic guanine monophosphate.
